# The Influence of Language Style and Brand Name on Crowdfunding Performance of Environmental Protection Enterprises

**DOI:** 10.1155/2022/6603923

**Published:** 2022-06-24

**Authors:** Qiong Sun, Jingjing Jiang, Jie Hu

**Affiliations:** Beijing Union University, Management College, Beijing, China

## Abstract

Crowdfunding, as an emerging phenomenon of enterprise after entrepreneurship financing, has maintained rapid and sustained growth in recent years. For crowdfunding environmental protection enterprises, one of the main challenges in financing is to reduce the uncertainty of public investors about the quality, management level, and products or services of crowdfunding projects. After reading the text of crowdfunding projects, the public investors have a subjective impression of the crowdfunding environmental protection projects, which determines the public investors' judgment on the risks and prospects of environmental protection projects and the willingness to invest. Therefore, the texts of crowdfunding projects are very important. In this paper, the data of 130 crowdfunding environmental protection projects on the Modian website are selected, and the ordinal logistic regression model is used. This paper explores the influence of language style in the description text and brand name in the title text on crowdfunding performance.

## 1. Introduction

Crowdfunding allows crowdfunding companies to raise money from mass investors via the Internet [1]. A crowdfunding platform provides a new channel for crowdfunding enterprises to seek financial help from the crowd, and its financing effect determines the rise and fall of crowdfunding enterprises [2]. The key to the success of crowdfunding projects is to minimize the public investors' perception of crowdfunding risks through effective communication [3]. Since crowdfunding projects usually involve emerging technologies that have not been verified, products and services to be tested by the market, and market demands that have not been verified, the impression of public investors on crowdfunding projects is inevitably determined by their subjective judgment [4]. One of the most important factors affecting the subjective judgment of public investors is the text of crowdfunding projects [5]. Crowdfunding project text is a typical user-generated content. The sponsor of a crowdfunding project can describe the financing project in any kind of language style on the crowdfunding platform. The public investors make investment decisions through the evaluation and selection of the project. If the crowdfunding project reaches or exceeds the target amount within the set period, the financing is successful [1]. At the end of crowdfunding, the ratio between the amount raised and the target amount is called crowdfunding performance [6].

On the Internet, public investors' investment decisions on crowdfunding projects will be affected by the environment and information. Scholars mainly study the influencing factors of crowdfunding performance from the aspects of information interaction and communication, project text description, text quantity and accuracy, text emotional tendency, and investor participation motivation. As for the research on the influence of narrative content on financing activities, Aristotle's rhetorical triad provides the basis for the research on the language style of crowdfunding projects. Some scholars have explored language metaphor and language framework, but the research on the influence of language style on crowdfunding performance is still lacking to some extent. In addition, only some crowdfunding enterprises clearly emphasized the brand name in the title of their crowdfunding activities, and many crowdfunding projects did not reflect it. Although the importance of brand advantage has been proved in the context of advertising and product marketing, the relevance of brand name in crowdfunding activities is still unknown. The existing theories, ideas, and empirical strategies have laid a certain foundation for studying the impact of language style and brand name on crowdfunding performance, while the research on the internal influence mechanism between relevant variables is slightly weak.

1. The existing research results on the influencing factors of crowdfunding performance pay more attention to the information interaction and communication, text description, text volume and accuracy, text emotional tendency, investor participation motivation, and other aspects of crowdfunding projects and rarely study the impact of language style on crowdfunding performance from the perspective of language style.
2. There are still differences in the definition of the language style of crowdfunding projects in the Chinese context, and no unified classification has been formed. The existing research mainly focuses on the impact of narrative content on financing activities, and the research on the impact of language style on crowdfunding performance is still lacking to a certain extent.
3. Brand name belongs to the concept of marketing, and there are few studies on enterprise management, especially related to crowdfunding activities. Although the importance of brand advantage has been proved in the context of advertising and product marketing, there are few studies on the relevance of brand name reflected in the project title in crowdfunding activities.

Based on the uncertainty reduction theory, this study reveals the influence mechanism of language style and brand name on crowdfunding performance through theoretical analysis and empirical test, tests the interaction effect of brand name on language style on crowdfunding performance, and guides crowdfunding enterprises to write targeted crowdfunding project texts and put forward management suggestions. Specifically, it includes (1) accurately define the language style used by crowdfunding projects in the Chinese context; analyze the influence mechanism of language style and brand name on crowdfunding performance; test the interaction effect of brand name on language style and crowdfunding performance; (2) guide crowdfunding enterprises to write targeted crowdfunding project texts; put forward management strategies that help crowdfunding enterprises improve crowdfunding performance in the Internet era.

## 2. Research Hypothesis

### 2.1. Language Style

Parhankangas & Renko divided language styles into concrete language, concrete language, interactivity language, and low psychological distance language. They used computer coding and LIWC dictionary to conduct an empirical study on the relationship between crowdfunding language style and crowdfunding performance [7]. Based on the research results, combined with the Chinese context, this paper defines the previously mentioned four language styles creatively and intends to explore the impact of detailed language, refined language, interactive language, and low psychological distance language on crowdfunding performance.

#### 2.1.1. Detailed Language

The detailed language in the Chinese context is characterized by a detailed description of the object, which is characterized by a detailed and accurate description. For the public investors, the detailed language effectively reduces the uncertainty of the prospects of crowdfunding projects and enhances their confidence in crowdfunding [7]. Studies have shown that most of the investment decisions made by public investors are based on very limited information transmission, and the specific and effective communication brought by detailed language has become one of the important reasons to promote the performance improvement of crowdfunding. Therefore, this study assumes the following.

H1a: using detailed language in crowdfunding project description is conducive to improving crowdfunding financing performance.

#### 2.1.2. Refining Language

Chinese and English are different in expression. English pursues precise expression in its development process. English aesthetics is refined and precise, while Chinese aesthetics is redundant and refined [8]. English emphasizes form and realism, while Chinese emphasizes conciseness, rhyme, and beauty [9]. Li Yan (2012) pointed out when studying the language style of tourism advertising, some Chinese tourism advertising texts reflect the Chinese people's thinking mode of “parataxis,” the unique four character structure in advertising language, or the common situation of imitative coinage of new words, which impresses people and promotes consumers' purchase intention [10]. Therefore, this study hypothesized the following.

H1b: using refined language in crowdfunding project description can improve crowdfunding financing performance.

#### 2.1.3. Interactive Language

Interactive language can show a high degree of interaction with potential readers, such as the use of questions [11]. Language styles that can quickly establish interpersonal relationships and are attractive are generally highly interactive [12]. The ability of interactive language to meet the needs of interactionists is stronger [13]. Zhe found that the use of interactive language in sales promotion can increase customers' understanding of advertising content and improve their purchase intention [14]. Therefore, this study hypothesized the following.

H1c: using interactive language in crowdfunding project description is conducive to improving crowdfunding financing performance.

#### 2.1.4. Low Psychological Distance Language

Psychological distance refers to the degree to which an individual is close, accepted, or difficult to get along with another individual or group. In environmental protection enterprises, it can refer to the extent to which investors want to get away from the environment under discussion [15]. Some scholars have confirmed that when there are too many low psychological distance language descriptions, there will be a certain degree of information redundancy, which makes it more difficult for public investors to obtain useful information from a large number of text descriptions when browsing crowdfunding projects, which may lead to some negative emotions of public investors [16] to reduce investment willingness and affect crowdfunding performance. Therefore, this study assumes the following.

H1d: using low psychological distance language in crowdfunding project description is not conducive to improving crowdfunding financing performance.

### 2.2. Brand Name

The title of crowdfunding project is the primary concern of public investors. The brand name reflected in the title text may increase the public investors' cognition and emotional response to crowdfunding projects [17], arouse the public investors' good attitude and response to crowdfunding activities [18], and reduce the perceived risk of public investors on the performance and quality of crowdfunding projects. Some crowdfunding projects cobranded with well-known brands are likely to have spillover effects [19]. It has aroused positive comments from the public investors. Therefore, this study assumes the following.

H2: brand name in the title is conducive to improving crowdfunding performance.

### 2.3. The Interactive Effect of Language and Brand Name

As the embodiment of brand name may increase the attention of public investors and lead to the change of public investors' attitude towards crowdfunding projects, based on hypothesis H1a to hypothesis h1d and hypothesis H2, this study assumes that there is interaction effect between brand name and the four language styles mentioned above, which positively affects crowdfunding financing performance.

  H3a: brand name has a positive impact on the relationship between detailed language and crowdfunding performance.
  H3b: brand name has a positive impact on refining language and crowdfunding performance.
  H3c: crowdfunding has a positive effect on brand performance.
  H3d: brand name has a negative impact on the relationship between low psychological distance language and crowdfunding performance.

Based on the previously mentioned theoretical background and research assumptions, the theoretical model of this paper is abstractly expressed in Figure 1.

## 3. Collection and Processing of Research Data

### 3.1. Data Source and Variable Selection

The initial sample of this study is from Motian, a well-known crowdfunding website in China. According to the following criteria for sample screening, (1) the project status is “completed,” (2) food products, scientific and technological products, and design products, and (3) no data are missing. Finally, 3506 sample sentences were screened from 130 effective crowdfunding projects, and the time span was from December 30, 2018, to December 20, 2021.

#### 3.1.1. Explained Variables

The explanatory variable in this study is crowdfunding performance, which is measured by the ratio of the amount raised by the project and the target amount at the end of crowdfunding [6]. The performance of crowdfunding financing truly reflects the financing effectiveness of crowdfunding projects.

#### 3.1.2. Explanatory Variables

*(1) Language style*. The core explanatory variables of this study are four language styles: detailed language, refined language, interactive language, and low psychological distance language. Chinese text structure is more complex than English. Under the interaction of phonology, syntax, semantics, and other elements, Chinese language has more complex characteristics than English [20]. Therefore, considering the actual situation of the data in this study, we choose the way of manual coding to get the language style corpus [21]. The four language styles are described in Table 1.

*(2) Brand name*. Virtual variables 1 and 2 indicate whether the brand name is reflected in the title text; 1 indicates that the brand name is not reflected in the title text, and 2 indicates that the brand name is reflected in the title text.

#### 3.1.3. Control Variables

Five control variables are selected in this study: (1) the target amount of financing; (2) video introduction; (3) unlocking the number of welfare files; (4) duration; (5) number of updates.

### 3.2. Sample Descriptive Analysis

On the basis of consulting relevant literature, combined with theory and practice, the four language styles (brand names, crowdfunding performance, and control variables) are classified and graded. Details are illustrated in Table 2.

## 4. Empirical Test and Result Analysis

### 4.1. Main Effect Test

#### 4.1.1. Model Applicability and Fitting Test

The applicability of ordered logistic model is verified by parallelism test [22]. Set the main effect test as model 1, and the parallelism test results show that *p* = 0.872 > 0.05, indicating that the results of this study are meaningful. The results of fitting test showed that the chi square value of model 1 was 70.115, *p* < 0.001; Pearson chi square value is 350.422, *p*=0.439. The deviation chi square value is 213.124, *p*=1. The previously mentioned test results show that the model can well explain the effect of language style and brand name on crowdfunding performance.

#### 4.1.2. Analysis of Model Results

The results of ordinal logistic regression are shown in Table 3.

1. The estimated values of regression coefficients for the number of detailed words in *X*_1_ = 1 and *X*_1_ = 2 are −1.718 and −1.457, respectively, and the OR values are 0.179 and 0.233. The data are significant at the level of 0.05. This shows that the use of less detailed language (1–379 words) in the description of crowdfunding projects significantly inhibits the improvement of crowdfunding financing performance. With the increase of the number of detailed language words, the OR value gradually increases. The estimated value of the regression coefficient of the number of detailed language words at *X*_1_ = 3 is −1.222, and the corresponding OR value is 0.295. The data is significant at the level of 0.1, indicating that with the increase of the number of detailed language words [23], the information of crowdfunding projects is fully received by public investors, and the negative effect on crowdfunding financing performance is gradually weakened. H1a is supported.
2. When the refined language (*X*_2_ = 1) is not used in crowdfunding project description, the data is not significant. When the number of refining words is between 1 and 34 words (*X*_2_ = 2), the estimated regression coefficient is 2.067, and the OR value is 7.901 > 1, which indicates that the use of appropriate refining language in crowdfunding project description can promote the investment willingness of public investors and significantly improve the performance of crowdfunding financing. With the increase of refining language words (35 words or more) in project description, crowdfunding performance is no longer improved, which indicates that using too much refined language may weaken the professionalism of crowdfunding projects. H1b is supported.
3. Interactive language is not significant in the data of *X*_3_ = 1, Xx_3_ = 2 and *X*_3_ = 3, so H1c is rejected. This may be because the interactive language may leave an abstract or general impression on the public investors, who may be more inclined to receive clear information.
4. When *X*_4_ = 1 and *X*_4_ = 2, the number of words in low mental distance language is not significant, which shows that when the number of words in the language of low psychological distance in the description of the crowdfunding project is less than 95 words, the public investors' evaluation of the development potential of the crowdfunding project and their investment willingness will not be affected, and the crowdfunding financing performance will not be significantly affected. When the number of words in low psychological distance language is *X*_4_ = 3, the estimated value of regression coefficient is 0.238, the OR value is 0.238 < 1, and the data is significant at the level of 0.05, which is close to the level of 0.01, which indicates that low psychological distance language is an obstacle to the financing performance of crowdfunding. When the number of words in low psychological distance language in the text of crowdfunding projects is too large (≥95 words), a certain degree of information redundancy will occur. It makes it more difficult for mass investors to obtain useful information from a large number of text descriptions when evaluating crowdfunding projects, affects investment willingness, and significantly inhibits crowdfunding financing performance. H1d is supported.
5. In terms of brand name, the estimated regression coefficient of *X*_5_ = 1 is −1.796, and the OR value is 0.166, *p* < 0.001, indicating that if the title text of the crowdfunding project does not reflect the brand name, it will significantly inhibit the crowdfunding financing performance. H2 is supported. This may be because the brand name reflected in the title can attract the attention of mass investors [24], convey the positive brand attitude of crowdfunding products to mass investors, and enhance their willingness to invest.

### 4.2. Interaction Effect Test

#### 4.2.1. Model Applicability and Fitting Test

Models 2∼4 are used to test the hypotheses H3a∼H3d.

The significances of models 2∼5 are 1, 0.810, 0.734, and 0.849, respectively, indicating that the models pass the parallelism test. The results of fitting degree test show the following.

The chi square value of model 2 is 70.514, *p* < 0.001; Pearson chi square value is 340.752, *p*=0.554; chi square deviation is 212.725, *p*=1.

The chi square value of model 3 is 70.672, *p* < 0.001; Pearson chi square value is 368.176, *p*=0.208*p*=0.208; chi square value of deviation is 212.566, *p*=1.

The chi square value of model 4 is 71.059, *p* < 0.001; Pearson chi square value is 348.007, *p*=0.520*p*=0.520; chi square value of deviation is 214.952, *p*=1.

The chi square value of model 5 is 76.197, *p* < 0.001; Pearson chi square value is 336.306, *p*=0.606; chi square value of deviation is 207.042, *p*=1.

The previously mentioned test results show that models 2∼4 can well explain the interaction effect.

#### 4.2.2. Analysis of Model Results

The results of ordinal logistic regression are shown in Table 4.

The results in Table 4 show that the regression coefficients of brand name and detailed language, refined language, and interactive language are not significant, so there is no interaction effect between brand name and detailed language, and the hypotheses H3a∼H3c are supported.

When the language interaction level of brand name and low psychological distance is *X*_11_ = 1, the data is not significant. When the interaction level is *X*_11_ = 2, the estimated regression coefficient was −2.06, and the OR value is 0.127 < 1, and the data is significant at the level of 0.05. When the interaction level is *X*_11_ = 3, the data is not significant. Compared with the regression results in Table 4, the data with *X*_4_ = 2 are significantly higher at the level of 0.05 and close to 0.01 in model 1, The OR value increased from 0.238 of model 1 to 0.657 of model 5. All these indicate that under the influence of brand name, the inhibition effect of low psychological distance language on crowdfunding financing performance is alleviated; that is, the brand name has a negative impact on the relationship between low psychological distance language and crowdfunding financing performance, and H3d is supported.

## 5. Core Conclusions and Management Suggestions

The core conclusions of this study are as follows.

1. The use of detailed language, refined language, and low psychological distance language in project description text can significantly affect crowdfunding performance. When the number of words is short, the performance of crowdfunding is significantly lower than that of words. Interactive language has no effect on crowdfunding performance.
2. Brand name in crowdfunding project title has a significant positive impact on crowdfunding performance. Brand name can reduce the perceived risk of public investors on crowdfunding projects, arouse the public investors' good attitude and response to crowdfunding projects, and enhance their investment willingness.
3. Brand name significantly negatively moderates the effect of low psychological distance language on crowdfunding performance but has no significant effect on detailed language, refined language, and interactive language.

According to the research conclusion, this study puts forward the following suggestions for the crowdfunding environmental protection enterprises to write crowdfunding project texts.

1. The detailed language should be used as much as possible in the description of crowdfunding projects, and the number of words should be more than 189 words, so as to fully demonstrate the credibility of crowdfunding projects, enable public investors to effectively evaluate the development potential of crowdfunding projects, reduce the risk perception of public investors, and make crowdfunding projects achieve higher financing performance.
2. In the description of crowdfunding projects, the number of refined words should be controlled between 1 and 34 words, so as to impress the public investors, enhance the investment willingness of the public investors, and help to obtain high crowdfunding financing performance. However, excessive use of refined language can weaken the professionalism of crowdfunding projects.
3. The low psychological distance language with too many words should not appear in the description of crowdfunding projects. When the number of words of low psychological distance in crowdfunding project description reaches 96 words or more, it increases the burden of public investors to obtain useful information and significantly inhibits crowdfunding financing performance.
4. Attention should be paid to the expression of brand name in the title of crowdfunding projects. The correct expression of the brand name in the title can arouse the attention of the public investors, stimulate the positive evaluation of the crowdfunding projects, stimulate the public investors to have brand association, and promote the crowdfunding financing performance. In addition, the empirical test results of this study show that, under the influence of brand name, brand name plays an important role. The inhibition effect of low psychological distance language on crowdfunding performance has been alleviated. Therefore, if the crowdfunding environmental protection enterprises inevitably use too many low psychological distance language (95 words and above) in the crowdfunding project description, we can consider to reflect the brand name in the title to alleviate the inhibition effect of low psychological distance language on crowdfunding financing performance.

## Figures and Tables

**Figure 1:** The theoretical model.

**Table 1:** Description of four language styles.

Variable	Variable description	Give an example
Detailed language	Describe the object in detail: detailed and accurate.	A real flower cake is a real flower cake.
Succinct language	Use refined adjectives or professional terms to describe an item or brand: classical poetry or refined sentences.	A successful boiled fish tastes smooth and tender, with bright red eyes and faint fish flesh,
Interactive language	A series of interactive languages such as questions, rhetorical questions, and invitations.	Let's drink with our favorite characters in the dream of red mansions!
Low psychological distance language	Language that brings psychological distance closer. It is manifested in the density of emotion and attitude.	Shh! This is our beautiful little secret∼

**Table 2:** Variable classification and sample description.

Category	Variable	Variable grading	Number of samples	Proportion (%)	Mean value
Dependent variable	Crowdfunding performance	1 = financing failure (crowdfunding performance <100%)	17	13.08	438.68%
		2 = low crowdfunding financing performance (100% ≤ crowdfunding financing performance <500%)	76	58.46	
		3 = medium crowdfunding financing performance (500% ≤ crowdfunding financing performance <1000%)	26	20	
		4 = high crowdfunding financing performance (crowdfunding financing performance ≥1000%)	11	8.46	

Independent variable	Detailed language	1 = 1–189 words	34	26.15	358.98 words
		2 = 190–379 words	46	35.38	
		3 = 380–569 words	30	23.08	
		4 = >569 words	20	15.38	
	Succinct language	1 = 0 words	60	46.15	52.05 words
		2 = 1–34 words	13	10	
		3 = 35–69 words	23	17.69	
		4 = >69 words	34	26.15	
	Interactive language	1 = 0 words	72	55.38	15.8 words
		2 = 1–59 words	49	37.69	
		3 = 60–119 words	6	4.62	
		4 = >119 words	3	2.31	
	Low psychological distance language	1 = 0 words	10	7.69	237.48 words
		2 = 1–94 words	39	30	
		3 = 95–189 words	22	16.92	
		4 = >189 words	59	45.38	
	Brand name	1 = no brand attention	45	34.62	
		2 = brand attention	85	65.39	

Control variable	Update times	1 = 1–9 times	100	76.92	6.67 times
		2 = 10–19 times	26	20	
		3 = >19 times	4	3.08	
	Duration	1 = 1–31 days	87	66.92	30.72 days
		2 = 32–62 days	36	27.69	
		3 = >62 days	7	5.38	
	Video introduction	1 = no video introduction	77	59.23	
		2 = with video introduction	53	40.77	
	Number of unlock benefit files	1 = 0 gear	28	21.54	46
		2 = 1–4 gears	87	66.92	
		3 = >4th gear	15	11.54	
	Financing target amount	1 = ≤20000 yuan	112	86.15	14667.87 yuan
		2 = 20001–40000 yuan	8	6.15	
		3 = >40000 yuan	10	7.69	

**Table 3:** Estimated values of main effect test parameters.

Variable			Coefficient	Standard error	Wald	Significance	OR value
Dependent variable	Crowdfunding performance	*Y* = 1 (unfinished)	−6.042^*∗∗∗*^	2.123	8.1	0.004	0.002^*∗∗∗*^
		*Y* = 2 (low financing performance)	−1.749	2.066	0.716	0.397	0.174
		*Y* = 3 (medium financing performance)	0.253	2.059	0.015	0.902	1.288

Independent variable	Detailed language Succinct language	*X*_1_ = 1 (1–189 words)	−1.718^*∗∗*^	0.664	6.7	0.01	0.179^*∗∗*^
		*X*_1_ = 2 (190–379 words)	−1.457^*∗∗*^	0.627	5.395	0.02	0.233^*∗∗*^
		*X*_1_ = 3 (380–569 words)	−1.222^*∗*^	0.672	3.308	0.069	0.295^*∗*^
		*X*_1_ = 4 (>569 words)	0^a^				
		*X*_2_ = 1 (0 words)	−0.329	0.52	0.4	0.527	0.720
		*X*_2_ = 2 (1–34 words)	2.067^*∗∗∗*^	0.746	7.679	0.006	7.901^*∗∗∗*^
		*X*_2_ = 3 (35–69 words)	0.679	0.628	1.17	0.279	1.972
		*X*_2_ = 4 (>69 words)	0^a^				
	Interactive language	*X*_3_ = 1 (0 words)	−1.078	1.418	0.578	0.447	0.340
		*X*_3_ = 2 (1–59 words)	−1.618	1.403	1.329	0.249	0.198
		*X*_3_ = 3 (60–119 words)	−0.287	1.66	0.03	0.863	0.751
		*X*_3_ = 4 (>119 words)	0^a^				
	Low psychological distance language	*X*_4_ = 1 (0 words)	−1.138	0.943	1.457	0.227	0.320
		*X*_4_ = 2 (1–94 words)	0.152	0.515	0.087	0.768	1.164
		*X*_4_ = 3 (95–189 words)	−1.436^*∗∗*^	0.605	5.645	0.018	0.238^*∗∗*^
		*X*_4_ = 4 (>189 words)	0^a^				
	Brand name	*X*_5_ = 1 (no brand name)	−1.796^*∗∗∗*^	0.489	13.521	<.001	0.166^*∗∗∗*^
		*X*_5_ = 2 (with brand name)	0^a^				

Control variable	Update times	*X*_6_ = 1 (1–9 times)	−3.191^*∗∗∗*^	1.18	7.319	0.007	0.041^*∗∗∗*^
		*X*_6_ = 2 (10–19 times)	−0.564	1.17	0.232	0.63	0.569
		*X*_6_ = 3 (>19 times)	0^a^				
	Duration	*X*_7_ = 1 (1–31 days)	2.001^*∗*^	1.038	3.713	0.054	7.396^*∗*^
		*X*_7_ = 2 (32–62 days)	1.132	1.016	1.242	0.265	3.102
		*X*_7_ = 3 (>62 days)	0^a^				
	Video introduction	*X*_8_ = 1 (no introduction)	−0.5	0.407	1.509	0.219	0.607
		*X*_8_ = 2 (with video introduction)	0^a^				
	Number of unlock benefit files	*X*_9_ = 1 (0 gear)	−1.662^*∗∗*^	0.75	4.912	0.027	0.190^*∗∗*^
		*X*_9_ = 2 (1st−4th gear)	−0.354	0.616	0.33	0.566	0.702
		*X*_9_ = 3 (>4th gear)	0^a^				
	Financing target amount	*X*_10_ = 1 (≤20000 yuan)	2.141^*∗∗*^	0.93	5.302	0.021	8.508^*∗∗*^
		*X*_10_ = 2 (20001–40000 yuan)	0.023	1.233	0	0.985	1.023
		*X*_10_ = 3 (>40000 yuan)	0^a^				

① The data are marked with ^*∗*^ at 0.1 level, ^*∗∗*^ at 0.05 level, and ^*∗∗∗*^ at 0.01 level; ^*∗∗∗*^② ^a^this parameter is redundant, so it is set to zero.

**Table 4:** Estimated values of interaction effect test parameters.

variable			Model 2		Model 3		Model 4		Model 5	
			Coefficient	OR value	Coefficient	OR value	Coefficient	OR value	Coefficient	OR value
Dependent variable	Crowdfunding performance	*Y* = 1 (unfinished)	−6.158^*∗∗∗*^	0.002^*∗∗∗*^	−6.297^*∗∗∗*^	0.002^*∗∗∗*^	−6.017^*∗∗∗*^	0.002^*∗∗∗*^	−6.708^*∗∗∗*^	0.001^*∗∗∗*^
		*Y* = 2 (low financing performance)	−1.864	0.155	−1.987	0.137	−1.709	0.181	−2.265	0.104
		*Y* = 3 (medium financing performance)	0.151	1.163	0.015	1.015	0.301	1.351	−0.202	0.817

Independent variable	Detailed language	*X*_1_ = 1 (1–189 words)	−1.442	0.236	−1.792^*∗∗∗*^	0.167^*∗∗∗*^	−1.655^*∗∗*^	0.191^*∗∗*^	−1.645^*∗∗*^	0.193^*∗∗*^
		*X*_1_ = 2 (190–379 words)	−1.054	0.349	−1.517^*∗∗*^	0.219^*∗∗*^	−1.393^*∗∗*^	0.248^*∗∗*^	−1.223^*∗*^	0.294^*∗*^
		*X*_1_ = 3 (380–569 words)	−0.923	0.397	−1.329^*∗*^	0.265^*∗*^	−1.184^*∗*^	0.306^*∗*^	−1.047	0.351
		*X*_1_ = 4 (>569 words)	0^a^		0^a^		0^a^		0^a^	
	Succinct language	*X*_2_ = 1 (0 words)	−0.336	0.715	−0.165	0.848	−0.292	0.747	−0.418	0.658
		*X*_2_ = 2 (1–34 words)	2.058^*∗∗∗*^	7.830^*∗∗∗*^	2.202^*∗∗*^	9.043^*∗∗*^	2.002^*∗∗∗*^	7.404^*∗∗∗*^	2.387^*∗∗∗*^	10.881^*∗∗∗*^
		*X*_2_ = 3 (35–69 words)	0.667	1.948	0.789	2.201	0.672	1.958	0.575	1.777
		*X*_2_ = 34 (>69 words)	0^a^		0^a^		0^a^		0^a^	
	Interactive language	*X*_3_ = 1 (0 words)	−1.077	0.341	−1.085	0.338	−0.722	0.486	−1.614	0.199
		*X*_3_ = 2 (1–59 words)	−1.599	0.202	−1.544	0.214	−1.061	0.346	−2.337	0.097
		*X*_3_ = 3 (60–119 words)	−0.34	0.712	−0.198	0.820	−0.243	0.784	−1.026	0.358
		*X*_3_ = 4 (>119 words)	0^a^		0^a^		0^a^		0^a^	
	Low psychological distance language	*X*_4_ = 1 (0 words)	−1.128	0.324	−1.165	0.312	−1.107	0.331	−0.435	0.647
		*X*_4_ = 2 (1–94 words)	0.189	1.208	0.256	1.292	0.084	1.088	1.252	3.497
		*X*_4_ = 3 (95–189 words)	−1.395^*∗∗*^	0.248^*∗∗*^	−1.461^*∗∗*^	0.232^*∗∗*^	−1.497^*∗∗*^	0.224^*∗∗*^	−0.42	0.657
		*X*_4_ = 4 (>189 words)	0^a^		0^a^		0^a^		0^a^	
	Brand name	*X*_5_ = 1 (without brand name)	−1.727^*∗∗∗*^	0.178^*∗∗∗*^	−1.704^*∗∗∗*^	0.182^*∗∗∗*^	−1.855^*∗∗∗*^	0.156^*∗∗∗*^	−1.294^*∗∗*^	0.274^*∗∗*^
		*X*_5_ = 2 (reflecting brand name)	0^a^		0^a^		0^a^		0^a^	

Control variable	Update times	*X*_6_ = 1 (1–9 times)	−3.155^*∗∗∗*^	0.043^*∗∗∗*^	−3.221^*∗∗∗*^	0.040^*∗∗∗*^	−3.154^*∗∗∗*^	0.043^*∗∗∗*^	−2.9^*∗∗*^	0.055^*∗∗*^
		*X*_6_ = 2 (10–19 times)	−0.522	0.593	−0.621	0.537	−0.496	0.609	−0.282	0.754
		*X*_6_ = 3 (>19 times)	0^a^		0^a^		0^a^		0^a^	
	Duration	*X*_7_ = 1 (1–31 days)	2.04^*∗*^	7.691^*∗*^	1.971	7.178	1.978^*∗*^	7.228^*∗*^	2.384^*∗∗*^	10.848^*∗∗*^
		*X*_7_ = 2 (32–62 days)	1.11	3.034	1.047	2.849	1.085	2.959	1.38	3.975
		*X*_7_ = 3 (>62 days)	0^a^		0^a^		0^a^		0^a^	
	Video introduction	*X*_8_ = 1 (no video introduction)	−0.481	0.618	−0.474	0.623	−0.505	0.604	−0.516	0.597
		*X*_8_ = 2 (with video introduction)	0^a^		0^a^		0^a^		0^a^	
	Number of unlock benefit files	*X*_9_ = 1 (0 gear)	−1.601^*∗∗*^	0.202^*∗∗*^	−1.693^*∗∗*^	0.184^*∗∗*^	−1.756^*∗∗*^	0.173^*∗∗*^	−1.913^*∗∗*^	0.148^*∗∗*^
		*X*_9_ = 2 (1st−4th gear)	−0.351	0.704	−0.331	0.718	−0.44	0.644	−0.549	0.578
		*X*_9_ = 3 (>4th gear)	0^a^		0^a^		0^a^		0^a^	
	Financing target amount	*X*_10_ = 1 (≤20000 yuan)	2.054^*∗∗*^	7.799^*∗∗*^	2.211^*∗∗*^	9.125^*∗∗*^	2.264^*∗∗*^	9.621^*∗∗*^	2.371^*∗∗*^	10.708^*∗∗*^
		*X*_10_ = 2 (20001–40000 yuan)	−0.133	0.875	0.02	1.020	0.141	1.151	0.076	1.079
		*X*_10_ = 3 = (>40000 yuan)	0^a^		0^a^		0^a^		0^a^	

Interaction item	Brand name *x* detailed language	*X*_11_ = 1 (≤400)	−0.423	0.655						
		*X*_11_ = 2 (401−800)	−0.627	0.534						
		*X*_11_ = 3 (801–1200)	−0.256	0.774						
		*X*_11_ = 4 (>1200)	0^a^							
	Brand name *x* refined language	*X*_12_ = 1 (≤400)			−0.411	0.663				
		*X*_12_ = 2 (401–800)			−0.026	0.974				
		*X*_12_ = 3 (801–1200)			−0.898	0.407				
		*X*_12_ = 4 (>1200)			0^a^					
	Brand name *x* interactive language	*X*_13_ = 1 (≤40)					−0.372	0.689		
		*X*_13_ = 2 (41–80)					−0.7	0.497		
		*X*_13_ = 3 (81 = 120)					−1.356	0.258		
		*X*_13_ = 4 (>120)					0^a^			

	Brand name *x* low psychological distance language	*X*_14_ = 1 (≤200)						−1.969	0.140	
		*X*_14_ = 2 (201–400)							−2.06^*∗∗*^	0.127^*∗∗*^
		*X*_14_ = 3 (401–800)							−1.212	0.298
*X*_14_ = 4 (>800)								0^a^	

① The data are marked with ^*∗*^ at 0.1 level, ^*∗∗*^ at 0.05 level, and ^*∗∗∗*^ at 0.01 level; ^*∗∗∗*^② ^a^this parameter is redundant, so it is set to zero.

## Data Availability

The raw/processed data required to reproduce these findings cannot be shared at this time as the data also form part of an ongoing study.
